# Intelligent Diagnosis Method for New Diseases Based on Fuzzy SVM Incremental Learning

**DOI:** 10.1155/2022/7631271

**Published:** 2022-01-13

**Authors:** Shi Song-men

**Affiliations:** China Pharmaceutical University, Nanjing 211198, China

## Abstract

The diagnosis of new diseases is a challenging problem. In the early stage of the emergence of new diseases, there are few case samples; this may lead to the low accuracy of intelligent diagnosis. Because of the advantages of support vector machine (SVM) in dealing with small sample problems, it is selected for the intelligent diagnosis method. The standard SVM diagnosis model updating needs to retrain all samples. It costs huge storage and calculation costs and is difficult to adapt to the changing reality. In order to solve this problem, this paper proposes a new disease diagnosis method based on Fuzzy SVM incremental learning. According to SVM theory, the support vector set and boundary sample set related to the SVM diagnosis model are extracted. Only these sample sets are considered in incremental learning to ensure the accuracy and reduce the cost of calculation and storage. To reduce the impact of noise points caused by the reduction of training samples, FSVM is used to update the diagnosis model, and the generalization is improved. The simulation results on the banana dataset show that the proposed method can improve the classification accuracy from 86.4% to 90.4%. Finally, the method is applied in COVID-19's diagnostic. The diagnostic accuracy reaches 98.2% as the traditional SVM only gets 84%. With the increase of the number of case samples, the model is updated. When the training samples increase to 400, the number of samples participating in training is only 77; the amount of calculation of the updated model is small.

## 1. Introduction

The acceleration of the pace of modern life and the aggravation of the pollution of air, water, and other living resources cause the increase of incidence disease rate [1]. Although the construction of medical conditions has made great progress, it is still stretched in the face of such a large population base. Medical staff and patients are facing great pressure.

With the development of artificial intelligence technology, it has been widely used in various fields and achieved very good results [2–5]. In the medical field, intelligent diagnosis and treatment have become a powerful tool and a hot spot [6, 7]. Machine learning, with its powerful data processing and mining ability, has become the main research direction of intelligent diagnosis and treatment: neural network, Bayesian network, random forest, support vector machine, and other methods have been applied to the exploration of this problem [8–12]. Particularly with the advent of the era of big data, the deep learning method [13] shows strong advantages.

Although these methods are effective, high-precision, the treatment often needs a lot of data support. At present, there are many channels for data acquisition. However, people often ignore a problem: the diagnosis of new diseases, especially those with strong infectivity. Coronavirus disease 2019 (COVID-19), which broke out in December 2019, is a very typical example of virus pneumonia. In the early stage of new crown, if the disease cases can be diagnosed quickly and accurately, the difficulty and cost of disease control will be greatly reduced. Many artificial intelligence methods have been adopted to help diagnosis [14–19]. Reference [20] proposed a deep migration learning method based on DenseNet201 to judge whether the patient is infected with COVID-19. A convolutional neural network model based on a multitask learning model was proposed in Reference [21] to realize COVID-19 detection and refinement of patient severity. Wang and Wong [22] proposed a CNN network model based on ResNet (COVID net). The model predicts normal, bacterial infection, non-COVID-19 viral infection, and COVID-19 viral infection, the accuracy is higher than 80%, and the computational complexity is less than 250 million times of multiplication and addition. Narin et al. propose three different deep learning models based on ResNet50, Inception V3, and Inception-ResNet v2 [23] to detect COVID-19 from X-ray images. All these studies have achieved high diagnostic accuracy, but they are based on large sample conditions. However, the initial case samples are very few. In this paper, we analyze this problem and study the intelligent diagnosis in the early stage of new diseases with few case samples.

This problem faces two challenges: (1) there are few sample data; (2) after the disease develops, the new case samples are added and the diagnostic model needs to be updated. In the machine learning method, SVM can deal with the classification problem well under the condition of small samples. Therefore, this paper selects the SVM method to solve this problem and learns the newly collected case samples through incremental learning, constantly updates and improves the diagnostic model, and improves the diagnostic ability [11, 12]. However, every time the diagnostic model of standard SVM is updated, all samples need to be retrained, which costs a lot of storage and calculation. To solve this problem, many scholars have proposed some SVM incremental learning methods. These methods mainly include three ideas: support vector, Karush Kuhn Tucker (KKT) condition, and the geometric features [24–29]. From the perspective of support vector idea, only support vectors have an impact on the solution [25, 26], so we only need to pay attention to the support vector. From the perspective of geometric features [28, 29], all the support vectors are at the boundary of the classification hyperplane. On this basis, in this paper, we intend to find out the support vector set and boundary sample set related to the SVM model, abandon most samples, ensure the classification accuracy of the model, and reduce the cost of calculation and storage.

In actual cases, some disease symptoms are similar, which brings difficulties to diagnosis. These features often exist as noise points. SVM adopts the same punishment method for all data points in the training process, which makes the training model more sensitive to noise and outliers. This situation will be more obvious when the number of samples is relatively small. In the incremental learning method we intend to adopt, most of the samples will be omitted in the sample updating process. In this case, if the traditional SVM training diagnosis model is still used, once some noise points or outliers with large deviation appear in the new samples, it may lead to a large deviation of the classification hyperplane, resulting in the possibility of a significant decline in the diagnosis effect. In this case, it is necessary to reduce the sensitivity of noise points and outliers. Lin and Wang proposed fuzzy support vector machine (FSVM) by introducing fuzzy membership function into standard SVM [30]. By giving different penalties to different samples, the influence of these points is weakened and the classification accuracy is improved.

To sum up, to solve the limited number of samples in the initial stage of new diseases, SVM is adopted. As the new samples are collected, this paper updates the diagnosis model in real time through the incremental learning method of SVM. At the same time, in order to reduce the impact of noise points on the model, the fuzzy membership function is introduced. It is hoped that these methods can improve the accurate diagnosis of new diseases and improve the diagnostic accuracy.

The rest of this paper is organized as follows: Section 2 introduces the SVM incremental learning method; the sample updating and the calculation method of fuzzy membership are proposed. In Section 3, the effectiveness of the proposed algorithm is verified by the banana dataset. In Section 4, an intelligent diagnostic application analysis was conducted using COVID-19 data; we discuss and compare the outcomes by experiment and analysis. Finally, conclusions are drawn and future directions are discussed in Section 5.

## 2. SVM Incremental Learning Method

The key of intelligent diagnosis is classification. The SVM method has the advantages of fast solution speed and strong generalization ability in solving small sample, nonlinear, and high-dimensional problems [31]. This is in line with the data characteristics in the early stage of new diseases. In this paper, SVM is selected as the diagnosis algorithm to realize the accurate diagnosis in the early stage of new diseases.

### 2.1. The Classification Principle of SVM

Assumes that the sample space of the case is *S* = {(**x**_*i*_, *y*_*i*_)|**x**_*i*_ ∈ *R*^*n*^, *y*_*i*_ = ±1, *i* = 1, ⋯, *l*}, where **x**_*i*_ is the feature vector of the disease and *y*_*i*_ is the corresponding state identification value (1 represents the target disease, and -1 represents the nontarget disease). SVM classifies disease diagnosis into convex quadratic programming shown in

(1) $$\begin{array}{c} \begin{array}{cc} \min & \frac{1}{2}{\left\|w\right\|}^{2}+C\overset{l}{\underset{i=1}{\sum }}\xi_{i}\\ \text{s}.\text{t}. & y_{i}\left(w\cdot x_{i}+b\right)\geq 1-\xi_{i},\\ \xi_{i}\geq 0,\;i=1,2,\cdots ,l, \end{array} \end{array}$$

where **w** is the normal vector corresponding to the optimal classification hyperplane and *C* is the penalty factor. The greater the *C* value, the greater the penalty for misclassification samples. *ξ* is a relaxation variable, which represents the distance from the sample points between the classification boundaries to the respective classification boundaries. The dual problem of equation (1) is shown in

(2) $$\begin{array}{c} \begin{array}{cc} \underset{\alpha }{\max} & \overset{l}{\underset{i=1}{\sum }}\alpha_{i}-\frac{1}{2}\overset{l}{\underset{i,j=1}{\sum }}\alpha_{i}\alpha_{j}y_{i}y_{j}K\left(x_{i},x_{j}\right)\\ \text{s}.\text{t}. & \overset{l}{\underset{i=1}{\sum }}y_{i}\alpha_{i}=0,\\ 0\leq \alpha_{i}\leq C,\;i=1,2\cdots ,l, \end{array} \end{array}$$

where *α*_*i*_ is the Lagrange multiplier. When (**x**_*i*_, *y*_*i*_) satisfies the Karush Kuhn Tucker condition given in equation (3), the corresponding optimal solution of equation (2) is

(3) $$\begin{array}{c} \left\{\begin{array}{c} \alpha_{i}=0\Rightarrow y_{i}f\left(x_{i}\right)\geq 1,\\ 0<\alpha_{i}<C\Rightarrow y_{i}f\left(x_{i}\right)=1,\\ \alpha_{i}=C\Rightarrow y_{i}f\left(x_{i}\right)\leq 1. \end{array}\right. \end{array}$$

The samples that violate the KKT condition (corresponding *α*_*i*_ ≠ 0) constitute the SV set, and the diagnostic model trained by the full sample set is shown in

(4) $$\begin{array}{c} y=\mathrm{sgn}\left[\overset{l}{\underset{i=1}{\sum }}y_{i}\alpha_{i}K\left(x,x_{i}\right)+b\right]. \end{array}$$

From the discrimination results of equation (4), we can see that the SVM-based diagnosis model only relates to the support vector set (SV set). The SV set is equivalent to the complete set.

### 2.2. Training Sample Set Update

Through the analysis above, we can get that for the SVM diagnosis method, the model is only related to the SV set. This is also applicable in the sample updating process of incremental learning. In the training process, we can simplify the updating process as long as we find the SV set in advance. For the SVM classification, the intuitive geometric interpretation is shown in Figure 1.

In Figure 1, solid dots and hollow dots represent two types of samples, respectively; *H* is the optimal classification hyperplane; *H*_1_ and *H*_2_ are the classification boundary hyperplanes parallel to *H* and passing through the nearest samples in two classes. *Margin* is the interval between classification boundaries. The positions of the SV set are mainly concentrated on the classification boundary and between the two classification boundaries, that is, the points identified by the red “o” in the figure.

Since only SV sets contribute to the classification hyperplane, the non-SV samples should be deleted during model update, which can reduce the amount of computation. For the newly added samples, if all samples are outside the classification boundary, meaning all the new samples are non-SV, they have no contribution to the diagnostic model. The added samples between two classification boundaries are usually new SVs. Due to these new samples, the previous classification boundary will be deflected, which will make some original non-SV_S_ transform into SV_S_ [28]. According to the geometric distribution of SV, the samples that may be transformed to SV are usually distributed near the classification boundary. Therefore, when updating the model, we need to take these sample points into account in addition to the original SV set. In this way, we can divide the updated sample set into three parts: the new sample set *S*_*n*_, the original SV set, and the sample set *S*_*h*_ near the classification boundary.

The sample set near the classification boundary:

(5) $$\begin{array}{c} S_{h}=\left\{\left(x_{i},y_{i}\right)\left|\begin{array}{c} x_{i}\in R^{n},y_{i}=\pm 1,\\ 1<\overset{l}{\underset{i=1}{\sum }}y_{i}\alpha_{i}K\left(x,x_{i}\right)+b<c,i=1,\cdots ,l \end{array}\right.\right\} \end{array}$$

where *c* is a constant; the number of selected samples of *S*_*h*_ can be adjusted through the setting of *c*. The smaller *c* is, the smaller size of the updated *S*_*h*_. It can obtain faster training speed and simpler diagnostic model. However, it may lead to the loss of key information and reduce the diagnostic accuracy. On the contrary, the larger the size of the updated *S*_*h*_, the higher the accuracy will be obtained. For incremental learning of model update, the update speed is determined by the number of training samples involved in the update. The smaller the number of training samples, the faster the update speed. Here, we further cut the updated sample set: in the new sample set, we use equation (5) to find the boundary samples. When updating the diagnostic model, only three sets of *S*_*n*_, SV, and *S*_*h*_ need to be retrained.

### 2.3. Fuzzy Support Vector Machine

FSVM first assigns membership values to the samples in the training set according to their importance in classification. The training sample set after evaluation is *S*′ = {(**x**_1_, *y*_1_, *μ*_1_), (**x**_2_, *y*_2_, *μ*_2_), ⋯, (**x**_*l*_, *y*_*l*_, *μ*_*l*_)}. *μ*_*i*_ ∈ [*ε*, 1] is the fuzzy membership of (**x**_*i*_, *y*_*i*_); *ε* is a sufficiently small positive number. Training *S*′ with SVM, the optimization problem in equation (1) transforms into the optimization problem:

(6) $$\begin{array}{c} \begin{array}{cc} \min & \frac{1}{2}{\left\|w\right\|}^{2}+C\overset{l}{\underset{i=1}{\sum }}\mu_{i}\xi_{i}\\ \text{s}.\text{t}. & y_{i}\left(w\cdot x_{i}+b\right)\geq 1-\xi_{i},\\ \xi_{i}\geq 0, & i=1,2,\cdots ,l. \end{array} \end{array}$$

Compared with the standard SVM, FSVM uses weighted error measurement *μ*_*i*_*ξ*_*i*_ to reduce the *ξ*_*i*_ in classification to a certain extent. As the outliers and noise in the sample are often within the classification boundary and have large relaxation variable values, FSVM weakens the influence of outliers and noise by assigning them small fuzzy membership, so as to avoid overfitting and improve the generalization of the diagnostic model. The core problem of FSVM is to give different fuzzy membership degrees to different sample points. In this paper, the fuzzy membership is determined by the relationship between points, classification hyperplane, and classification boundary. The samples are divided into inside boundaries and outside boundaries. The samples outside the boundary can be considered as determined sample, and the fuzzy membership degree is set 1. If the sample points are misclassified, we give its fuzzy membership a very small value *ε* (here *ε* = 0.0001). The correctly classified samples between the boundaries are the samples that we should focus on. Consider the interval between the sample points and the optimal classification hyperplane. The farther the interval, the greater the probability that they belong to this category. The interval of the optimal classification hyperplane of sample points *m* can be expressed as

(7) $$\begin{array}{c} m=\left|\overset{l}{\underset{i=1}{\sum }}y_{i}\alpha_{i}K\left(x,x_{i}\right)+b\right|. \end{array}$$

The final fuzzy membership function is

(8) $$\begin{array}{c} \mu =\left|{\left(\frac{2}{{\left(m-1\right)}^{2}}-1\right)}^{-1}-1\right|. \end{array}$$

The function diagram of fuzzy membership function is shown in Figure 2.

The fuzzy membership function is constructed by the generalized bell membership function model. When *m* changes from 0 to 1, the first half *u* increases rapidly because it is close to the optimal classification hyperplane and away from the sample class; the latter half is close to the classification boundary, and the increase of value *u* tends to be gentle.

### 2.4. Diagnostic Process

The processing process of the intelligent diagnosis method based on FSVM incremental learning is shown in Figure 3.

Firstly, the initial model is established by the previously collected historical case database and is used to judge whether it is the target disease and give specific diagnosis and treatment suggestions; according to the recovery of patients, the misdiagnosed and missed cases in the initial diagnosis results are analyzed. After being identified by experts, they are input into the historical sample database as incremental samples. When the incremental samples accumulate to a certain number, the model update program is triggered; in the model updating stage, the SV set and boundary sample set are extracted from the historical sample database according to the diagnosis results of historical samples, and they are added together with the boundary samples and boundary samples in the new sample set as a new training sample set, and a new diagnosis model is obtained by giving different fuzzy membership degrees to different samples for FSVM training. The intelligent diagnosis system incorporated into the model update forms a closed-loop self-learning system, which is conducive to the continuous correction and improvement of the diagnosis model and enhances the SVM's ability to diagnose new diseases.

## 3. Algorithm Verification

In order to verify the effectiveness of the proposed method in this paper, we select the typical two-dimensional nonlinear separable dataset banana dataset in benchmark dataset [32] and verify the performance of the algorithm by updating the classification samples of the dataset and analyzing the classification results. The experimental environment is Xeon (R) 3.3G CPU, 8G memory, Windows 7 system, and MATLAB 2018b. RBF kernel function is selected for SVM training. Its parameters are determined by cross-validation and grid search method and *c* set to 1.5.

Firstly, we analyze the sample update results of the algorithm.  Figure 4 shows the classification of the banana dataset (the initial training set includes 150 sample points of positive and negative classes) under initial training. The purple, green, and yellow contours in Figure 4 represent the positive class sample classification boundary, the optimal classification hyperplane, and the negative class classification boundary, respectively. “o” represents the set of support vectors, and “□” represents the set of boundary samples found. From the figure, we can see that the support vector sets are distributed within and on the classification boundary, and the boundary sample sets are near the classification boundary. This verifies the previous analysis is correct. These samples contain all the classification boundary information.

Next, the rationality of the updated fuzzy membership function is verified. We added 50 positive and negative samples, respectively.  Figure 5 shows the updated dataset and their fuzzy membership. The red “o” point in the figure is all the updated sample sets (including the boundary sample set found earlier, support vector set, and new sample set after clipping). The size of “o” represents the value of fuzzy membership. It should be noted that for better display effect, the minimum size of “o” is set to the size of 8 labels in MATLAB. It can be clearly seen from the experimental results that the sample point “o” at the classification boundary is the largest. The closer the point between the two classification boundaries is to the optimal classification hyperplane, the smaller its value. In this way, their influence on the classification model can be reduced during training, and the misclassified sample points are the smallest, which means that they can be almost ignored during training. In this way, FSVM can improve the generalization of the classification model.

Finally, we analyze the classification performance of the updated classification model after adding new samples. Compare the nonupdated classification hyperplane, the SVM incremental learning updated model, and the classification model by adding fuzzy membership.  Figure 6 shows the classification results of the three methods. From the results, we can see that the classification model has changed after incremental learning. This is mainly because the addition of new training samples affects the original classification hyperplane after incremental learning. The newly obtained classification hyperplane is more accurate than the original classification hyperplane. Compared with the classification hyperplane obtained by the two update methods, FSVM can effectively reduce the impact of noise points and outliers by giving different penalty coefficients to different training samples. For example, as can be seen from the local amplification part in Figure 6, the optimal classification hyperplane is biased to the right due to the influence of two “.”. The FSVM can effectively modify the classification hyperplane and improve generalization.

Further, we continuously add the sample set to the training set, with each increase of 100 samples (positive class 50, negative class 50). The updated model is tested on banana_test_2. The specific classification accuracy results are shown in Table 1.

From the experimental results in Table 1, we can see that if there is no incremental learning, the accuracy of the classification model is only 86.4%. However, through incremental SVM learning, the model is continuously optimized with the update of the sample set, and finally, the classification accuracy of 89.8% is achieved. Through the introduction of fuzzy factor, the generalization of the model is further improved, and the classification accuracy can reach 90.4%. In the process of model updating, the size of training set will affect the training time and the timeliness of model updating. The proposed method in this paper can filter the initial samples and only select the support vector set and boundary sample set; the number of samples participating in the update is very small. So the update speed of the model is also relatively fast.

## 4. Application Analysis of Intelligent Diagnosis

In order to verify the effectiveness of the proposed algorithm, an intelligent diagnostic application analysis was conducted using COVID-19 data provided by our affiliated hospital. The dataset includes two types of samples: COVID-19 and non-COVID-19. The total number of samples was 571, including 357 non-COVID-19 and 212 COVID-19.

The sample includes a total of 37 features. The first two features are patient ID and category. Excluding these two-dimensional features, the remaining 35 dimensions are the features we use for diagnosis. Overall, it includes physiological features, biochemical examination results, and CT image characteristics. The physiological features include ambulatory blood pressure, pulmonary hypertension, heart rate, SpO_2_, body temperature, and respiratory rate. The biochemical examination mainly includes the following features: the number of white blood cells, the percentage of lymphocytes, creatine kinase, alanine aminotransferase, aspartate aminotransferase, high-sensitivity C-reactive protein, and erythrocyte sedimentation rate. The CT image features mainly include density, shape, lesion distribution, interstitial thickening, thickening of vascular bundle in the lesion, cord focus, and pleural effusion. From the overall data, the ratio of non-COVID-19 and COVID-19 is about 6 : 4. We assume that 100 groups of cases were collected in the initial stage, of which 60 groups are non-COVID-19 and 40 groups are COVID-19. The selection method is random. Incremental learning is performed every 100 samples. Finally, the remaining 171 groups were used as the sample set for the test. The experimental results are shown in Table 2.

From the experimental results, we can see that the diagnostic accuracy is gradually improved with the increase and improvement of the sample set, which is similar to the previous experiments on the banana dataset. In the initial sample set, there are only 100 cases; the diagnostic accuracy of the diagnostic model has reached 84.0%, which reflects the advantages of the SVM method in dealing with small samples. The classification accuracy of the same data trained by the BP neural network is only 74.6%, which is far lower than that of the SVM method. If incremental learning is not used to update the sample set and diagnostic model, the diagnostic accuracy of such model is far from enough, which means that more than 15% of patients will be misdiagnosed. When only the SVM method is used to update the model, the diagnostic accuracy has been greatly improved due to the new case samples, and the final diagnostic accuracy can reach 95.9%. However, the existence of wild points and noise points may reduce the generalization of the model. Through the fuzzy processing of these sample points, FSVM can effectively reduce their impact on the classification hyperplane of the model and improve the generalization. The experimental results show that the incremental learning model processed by FSVM can improve the diagnosis accuracy to 98.2% and further verify the advantages of FSVM incremental learning.

Another key problem to be considered in incremental learning is the update speed. With the increase of samples, if the update speed is too slow and does not have real-time performance, the whole incremental learning method will not be applied to practice. For SVM learning, the speed of training depends on the number of samples participating in training. If the updated training samples are not clipping, the storage and calculation cost of the system will get higher. The method proposed in this paper discards the useless sample points on the basis of the previous model.  Figure 7 shows the number of training samples trained by SVM without clipping and the number of training samples updated by the method in this paper. From the figure, we can see that without clipping, the number of samples gradually increases with the change of model update iteration and has reached 400 by the fourth update. The proposed method makes necessary selection every time, and the number of sample points is relatively stable. Even in the fourth generation, the number of samples participating in training is only 77. It can be seen that the method in this paper can greatly reduce the amount of calculation and ensure the efficiency of updating.

Next, we analyze the accuracy of the overall diagnosis of the model. Here, the confusion matrix is chosen to judge the binary classification problem. The confusion matrix is shown in Table 3.

According to Table 3, the recall rate and accuracy rate of the diagnostic model can be calculated as follows:

(9) $$\begin{array}{c} \text{recall rate}=\frac{\text{TP}}{\text{TP}+\text{FN}},\\ \text{accuracy rate}=\frac{\text{TP}}{\text{TP}+\text{FP}}. \end{array}$$

In the diagnostic problem, the recall rate can represent the proportion of correctly identified positive cases in all confirmed cases. This measures the recognition ability of the diagnostic model for new diseases. The accuracy rate is oriented to the training model, which represents the proportion of confirmed cases identified by the model. The two measure the diagnostic performance of the diagnostic model from different angles. We generally combine the two to draw precision-recall (PR) curves to investigate the diagnostic model. The PR curves under different samples and methods are shown in Figures 8 and 9.

When the PR curve is closer to the upper right, it indicates that the performance of the model is better. When comparing different models, if the PR curve of one model is completely covered by the PR curve of another model, it indicates that the performance of the latter is better than the former. From the experimental results in Figure 8, we can see that with the increase of samples and the update of the diagnostic model, the PR curve of the new diagnostic model gradually approaches to the right and up, and the PR curve updated each time can completely cover the previous curve, which also shows that the proposed FSVM incremental learning method can effectively improve the performance of the diagnostic model. From Figure 9, compared with the SVM without update and the SVM incremental method, the FSVM incremental learning method can also cover the other two methods, and the curve obtained is more upper right than the other two methods, which also shows that the FSVM incremental learning diagnosis method proposed in this paper can obtain better diagnosis effect.

## 5. Conclusion

The diagnosis of new diseases is a challenging problem in intelligent diagnosis and treatment with machine learning. In order to solve the problem of few sample cases, the SVM method is selected in this paper. At the same time, incremental learning is used to update the sample database and diagnostic model. Incremental learning is an important means to ensure that the knowledge-based intelligent diagnosis method can adapt to the increase of samples. According to the basic principle of the SVM method, this paper determines the sample set related to the model, mainly including support vector set, boundary sample set, and new sample set, in which boundary sample set solves the problem of support vector transformation. In order to solve the problem that the influence of noise points and outliers on the diagnosis results increases after the number of samples is reduced, the FSVM method is used in the process of model updating. Experiments show that the proposed method not only effectively simplifies the incremental training set but also effectively improves the training efficiency while ensuring the diagnosis accuracy. The addition of fuzzy membership also effectively improves the generalization of the model. The research of this paper can provide a new idea for the application of machine learning method in the field of intelligent medical diagnosis, especially in the early stage of new diseases and the real-time update of the diagnosis model. Future directions include continuing to improve sensitivity and accuracy for COVID-19 and other new disease infections as new data is collected, as well as extend the proposed method to risk stratification for survival analysis, predicting risk status of patients and so on.

## Figures and Tables

**Figure 1:** SVM classification diagram.

**Figure 2:** Fuzzy membership function.

**Figure 3:** Intelligent diagnosis process based on FSVM incremental learning.

**Figure 4:** The classification result of the banana dataset.

**Figure 5:** Updated set and fuzzy membership.

**Figure 6:** Results of FSVM incremental learning classification.

**Figure 7:** Size of FSVM incremental training sample.

**Figure 8:** The PR curve of FSVM incremental learning diagnosis.

**Figure 9:** The PR curve of FSVM incremental learning and other diagnosis methods.

**Table 1:** Comparison of classification accuracy of the banana dataset.

Training set		Test set	Classification accuracy (%)	
			SVM	FSVM
Initial set	Positive 150, negative 150	Banana_test_2	86.4	
Increment 1	Positive 50, negative 50		88.2	88.4
Increment 2	Positive 50, negative 50		88.6	89.1
Increment 3	Positive 50, negative 50		89.4	90.2
Increment 4	Positive 50, negative 50		89.8	90.4

**Table 2:** Diagnosis results.

Training set		Test set	Diagnostic accuracy(%)	
			SVM	FSVM
Initial set	Non 60, COVID-19 40	Non 118, COVID-19 53	84.0	
Incremental 1	Non 57, COVID-19 43		87.6	88.8
Incremental 2	Non 64, COVID-19 36		91.1	93.4
Incremental 3	Non 63, COVID-19 37		95.9	98.2

**Table 3:** Confusion matrix of diagnosis problem.

Predictive	Actual	
	COVID-19	Non-COVID-19
COVID-19	TP	FP
Non-COVID-19	FN	TN

## Data Availability

Data will be available from the corresponding author upon request.
